The article "Diagnostic Accuracy Rates of Appendicitis Scoring Systems for the Stratified Age Groups" was published in 2022. Journal: Emerg Med Int.

# Diagnostic Accuracy Rates of Appendicitis Scoring Systems for the Stratified Age Groups

**DOI:** 10.1155/2022/2505977

**Published:** 2022-10-31

**Authors:** Emre Gonullu, Zulfu Bayhan, Recayi Capoglu, Barış Mantoglu, Burak Kamburoglu, Tarık Harmantepe, Fatih Altıntoprak, Unal Erkorkmaz

**Affiliations:** ^1^Sakarya University, Faculty of Medicine, Department of Gastrointestinal Surgery, Serdivan, Sakarya, Turkey; ^2^Sakarya University, Faculty of Medicine, Department of General Surgery, Serdivan, Sakarya, Turkey; ^3^Sakarya University, Training and Research Hospital, Department of General Surgery, Serdivan, Sakarya, Turkey; ^4^Sakarya University, Faculty of Medicine, Department of Biostatistics, Serdivan, Sakarya, Turkey

## Abstract

**Background:**

Many scoring systems have been developed for acute appendicitis, which is the most common emergent disorder in surgical practice. Considering the physiological changes and chronic diseases occurring with advancing age, an applied scoring system may not produce the same score in similar patients in all age groups.

**Objectives:**

We aimed to compare the predictive values of scoring systems in different age groups.

**Methods:**

In this prospective study, the patients operated on in our clinic with a prediagnosis of acute appendicitis between March 2020 and March 2021 were included. We divided them into three age groups as 18–45 years (group 1), 46–65 years (group 2), and >65 years (group 3). We compared the scores of the nine acute appendicitis scoring systems most commonly used in the literature for these age groups.

**Results:**

A total of 203 patients were included in our study. The Alvarado scoring system yielded the most accurate results for group 1, whereas the Fenyo–Linberg scoring system was the most accurate system for group 2 and the Eskelinen scoring system for group 3.

**Conclusion:**

Age should be considered as a major parameter during the selection of the scoring system to be applied for patients with prediagnosis of acute appendicitis. Our study revealed the Alvarado and the Fenyo–Lindberg scoring systems as the most accurate systems for the differential diagnosis of appendicitis in the 18–45 and 46–65 years age groups, respectively. Although we found the Eskelinen scoring system as the most accurate one in the >65 years age group, the confidence intervals indicated that it may not be appropriate for use alone in this group.

## 1. Introduction

Acute appendicitis remains the most frequent disorder requiring an emergent surgical intervention worldwide and occurs approximately in one of 10 individuals during the life course [1]. Considering that acute appendicitis commonly occurs in young employed adults, it also has negative economic and social impacts [2, 3]. Although various studies have reported that the incidence of acute appendicitis remains higher in younger people, in particular, the males, acute appendicitis is no longer exclusively a disease of the youth in developed countries but also frequently seen in middle and advanced ages also [4–6].

Appendectomy is the most commonly performed abdominal surgery in general surgical practice. However, the negative appendectomy rates remain quite high (6.2–15.9%) despite the improved facilities and radiological examination methods [7, 8]. The abdominal surgical procedures, or a perforated appendix, can cause severe morbidities, such as recurrent episodes of intestinal obstruction due to intra-abdominal adhesions, ectopic pregnancy etc. [9, 10]. Thus, timely and accurate diagnosis is essential for the proper management [11, 12]. The most useful parameters for diagnosing acute appendicitis are the duration of abdominal pain, physical examination findings, and laboratory parameters. Various imaging methods are used to validate the prediagnosis [13]. Many clinical scoring systems (CSSs) using different parameters have been developed to predict acute appendicitis [14, 15]. The purpose of applying a CSS is to predict acute appendicitis and distinguish the patients who need medical treatment or needing an emergent surgery preventing the probable complications that may increase mortality and morbidity [1, 16]. CSSs may facilitate differential diagnosis reducing the unnecessary radiologic examinations and surgical explorations [17]. Many previous studies have compared the effectiveness of CSSs developed for acute appendicitis [13, 15]. Although the efficacy of these CSSs for the pediatric age group has been evaluated, no study has compared the efficiency of these scoring systems among adult age groups [18].

In the present study, we aimed to compare the predictive values of scoring systems in different age groups. We tested the hypothesis proposing that a CSS may not show consistency in terms of accuracy rate among the different stratified age groups.

## 2. Materials and Methods

This prospective study was approved by our institutional review board (approval no: 71522473/050.01.04/44). The study was conducted in a tertiary training and research hospital. We evaluated patients aged >18 years with a diagnosis of acute appendicitis operated on in our clinic between March 2020 and March 2021.

### 2.1. Exclusion Criteria

We excluded patients aged <18 years, pregnant patients, those who had given birth in the last 3 months, those with an existing malignancy, patients using steroids for any reason, immunosuppressed patients, COVID-19-positive patients, and patients with previous pelvic inflammatory disease.

### 2.2. Study Setting

An emergency medicine specialist evaluated patients who presented to the emergency department with abdominal pain. The general surgical assistant physician was consulted after requesting blood tests and ultrasound (US) from each patient with a suspected acute abdomen. Subsequently, the surgical assistant examined the patients, evaluated the tests, and consulted the on-duty surgeon. The on-duty consulting surgeon examined each patient within the first hour after the consultation. An abdominal computed tomography (CT) scan was performed in cases where there was doubt about the diagnosis. Following these examinations, the consulting surgeon hospitalized the patients with a preliminary diagnosis of acute abdomen. The emergency physician discharged the other patients or consulted with other departments. The general surgery assistant collected the variables required to calculate the scores for each system (RIPASA (Raja Isteri Pengiran Anak Saleha Appendicitis), Appendicitis Inflammatory Response (AIR), and the scoring systems of Tzanakis, Eskelinen, Ohmann, Lintula, Fenyo–Lindberg, and Karaman) used to predict acute appendicitis (Table 1) and calculated each patient's score for each scoring system. Regardless of the CSS result (the results were not disclosed to the surgeon), the consulting surgeon evaluated the patient's history, physical examination findings, and laboratory and radiological examination results, and an open or laparoscopic appendectomy procedure was performed if the patient was diagnosed with acute appendicitis. We defined the outcome of appendicitis according to the histopathological examination and recorded the histopathological examination results on the same datasheet to evaluate the accuracy of the CSSs for predicting acute appendicitis. We divided the patients into three age groups (18–45, 46–65, and >65 years). Statistical analyses were performed to compare the scoring systems between the groups.

### 2.3. Statistical Analysis

Descriptive analyses were performed to obtain information on the general characteristics of the study population. We used the Kolmogorov–Smirnov test to evaluate whether the distributions of numerical variables were normal. We used the independent-samples*t*-test and Kruskal–Wallis test to compare the numeric variables between the groups. The numeric variables are presented as mean ± standard deviation or median (Q1–Q3). Categorical variables were compared to the chi-square test, and are presented as counts and percentages. A *p* value <0.05 was considered significant. We used receiver operator characteristic curve analysis to identify the best cut-off values and assess the performance of the appendicitis test scores. Analyses were performed using SPSS statistical software (version 23.0; IBM Corp., Armonk, NY, USA).

## 3. Results

### 3.1. General Characteristics of the Patient Group

During the 1-year study period, 203 patients were evaluated. In total, 129 (63.5%) of these patients were male, and 74 (36.5%) were female. The ages of the patients were 18–83 (mean = 37 ± 16) years. A total of 149 patients (73.4%) were in the 18–45 years age group, 34 (16.7%) were in the 46–65 years age group, and 20 (9.9%) were in the >65 years age group. A total of 197 (97%) patients were native and 6 (3%) were foreign.

### 3.2. Patients with and without Appendicitis

Appendicitis was determined by histopathological examination in 180 of the 203 patients. The mean age of the patient group with appendicitis was 37.43 ± 16.71 years, while that of the patient group without appendicitis was 32.09 ± 17.50 years. A total of 118 (65.5%) patients with appendicitis were male and 62 (34.5) were female. In total, 176 (97.7%) patients with appendicitis were native, and 4 (2.3%) were foreign. No significant differences in age, gender, or nationality were observed between patients with and without appendicitis (*p*=0.67, 0.96, and 0.84, respectively). We observed appendicitis by US in 169 patients with appendicitis but could not detect appendicitis in 11 (sensitivity: 91.4%, specificity: 38.9%) (Table 2).

The pain relocation rate was significantly higher in the appendicitis group than in the group without appendicitis (53.6% vs. 34.8%, *p*=0.04).

The rate of decrease in bowel sounds on auscultation was higher in the appendicitis patient group than in the group without appendicitis (10% vs. 4%, *p*=0.004).

No significant differences were detected in white blood cell (WBC) count, C-reactive protein (CRP) level, or the polymorphonuclear leukocyte ratio (*p*=0.48, 0.22, 0.12, and 0.08, respectively) between patients with and without appendicitis, except that the WBC count in the 18–45 years age group was significantly higher in patients with than without appendicitis (14,950 ± 19,751 vs. 12,800 ± 3,248 *μ*l/ml, *p*=0.001).

### 3.3. Comparisons among the Three Age Groups

No significant differences in gender or nationality were observed among the three groups (*p*=0.811, 0.851, respectively).

A higher proportion of the 18–45 years group were admitted to the hospital at an early stage than in the other age groups (*n* = 86/149; 57.7%; *p*=0.04). The proportion of patients with abdominal pain onsetting in the periumbilical region that relocated to the right lower quadrant was significantly lower in the >65 years group than in the other two age groups (*n* = 15/20; 75%; *p*=0.02). No differences in any other complaints were observed among the groups (Table 2).

No significant differences in the physical examination findings were observed among the age groups.

The CRP level was significantly higher in the >65 years group than in the other two groups (86.8 (42.6–146.13) mg/L) (*p*=0.002). The leukocyte count was higher in the 18–45 years group than in the other two groups (14,600 (11,100–17,200) *μ*l/ml) (*p*=0.049). No differences in any other blood parameters or urinalysis were observed among the age groups. The rate of appendicitis detection by US was 91.3% (*n* = 136/149) in the 18–45 years age group, 91.2% (*n* = 31/34) in the 46–65 years group, and 90% (*n* = 18/20) in the >65 years group. Acute appendicitis was revealed radiologically in 41 (91%) of 45 patients evaluated by CT. However, the diagnosis of only 39 (94.2%) of these patients was confirmed by histopathological examination; appendicitis was not detected in the remaining 2 patients (4.8%).

Histopathological examination of the pathology specimens revealed that 88.7% (*n* = 180/203) of the patients had appendicitis, and 11.3% (*n* = 23/203) did not. The appendicitis rates on histopathological examination were 87.2% (130/149), 94.1% (32/34), and 90% (18/20) in the 18–45, 46–65, and > 65 years age groups, respectively (Table 3).

### 3.4. Accuracy of the Scoring Systems

When all patients were analyzed together, the Fenyo–Lindberg (area under the curve (AUC): 05980; positive predictive value (PPV): 93%; negative predictive value (NPV): 17%; sensitivity: 60%; specificity: 65%) and Alvarado (AUC: 0.62; PPV: 92%; NPV: 25%; sensitivity: 81%; specificity: 47%) scoring systems were more accurate for predicting appendicitis than the other CSSs. The most accurate scoring systems in the 18–45 years group were the Alvarado (AUC: 0.66; PPV: 92%; NPV: 29%; sensitivity: 83%; specificity: 47%) and Fenyo–Lindberg CSS (AUC: 0.65; PPV: 92%; NPV: 21%; sensitivity: 65%; specificity: 63%) CSSs. The most accurate scoring systems in the 46–65 years group were the Fenyo-Linberg (AUC: 0.68; PPV: 100%; NPV: 10%; sensitivity: 46%; specificity: 100%) and Karaman (AUC: 0.62; PPV: 100%; NPV: 8%; sensitivity: 31%; specificity: 100%) CSSs. The most accurate scoring systems in the >65 years group were the Eskelinen (AUC: 0.61; PPV; 100%; NPV: 18%; sensitivity: 50%; specificity: 100%) and Tzanakis (AUC: 0.52; PPV; 92%; NPV; 14%; sensitivity; 66%; specificity: 50%) CSSs (Table 4).

## 4. Discussion

The diagnosis of appendicitis can be made with 75% certainty via physical examination and based on the complaints of patients [13]. However, we did not find any significant differences in physical examination findings on admission between patients with and without appendicitis, except for bowel sounds on auscultation and relocated pain. To perform the auscultation, the stethoscope is placed over the abdomen skin and the sounds produced by intestinal peristalsis are listened. However, the auscultation is a subjective examination method. It provides information about the presence of peritonitis but could not be used in the differential diagnosis. In their recent clinical study, Zaborski et al. suggested that the evaluation of the structure of bowel sounds might enable the use of bowel sounds when making a differential diagnosis [19]. Physical examination findings and laboratory parameters are frequently reported in the literature as important factors for diagnosing acute appendicitis in patients aged 20–40 years who do not have a chronic disease or history of regular medication use or pregnancy [13]. Chronic medication use in the elderly and changes in pain tolerance with age may underlie the differences in physical examination findings and blood parameters between age groups, and the variations in diagnostic parameters, rendering the diagnosis of acute appendicitis challenging [20].

Abdominal US, physical examination findings, and laboratory parameters have different weights among scoring systems, and some parameters are not included in all systems. Therefore, it should not be expected that CSSs have the same predictive value in every age group.

Abdominal CT  screening increases the accuracy of acute appendicitis diagnosis, and high sensitivity and specificity can be achieved (98%). However, a CT scan is not routinely recommended for diagnosing acute appendicitis due to known disadvantages including radiation exposure, high cost, and unsuitability for pregnant women [21–24]. CT is more beneficial in complex cases where US is inadequate. Furthermore, the 2020 World Society of Emergency Surgery (WSES) guidelines recommend that CT be performed only in cases of negative US findings; this will reduce the rate of CT by 50%. They recommended this strategy in patients with suspected appendicitis [3]. In our study, while US was performed in all patients during the preoperative period, CT was used in only 22.1% of patients, in accordance with the strategy proposed by the WSES. Our negative appendectomy rate was 11.3%, which is consistent with the literature [7].

Considering the high sensitivity and specificity of US for diagnosing acute appendicitis, the Tzanakis CSS, which uses US as a criterion, was expected to be more accurate in all age groups [21, 25]. However, this will only apply if all US examinations are performed under ideal conditions, and by experienced operators. Tzanakis et al. reported that US produced a false-negative rate of 24% for diagnosing appendicitis in the 2005 study in which they introduced their score [21]. Various studies have demonstrated that numerous factors affect the performance of the radiologist, such as the daily patient load, clinical experience, and consultations outside of working hours [15, 26]. Moreover, the importance of US in the Tzanakis score (6 of 15 points, 40%) means that the radiologist's performance is the most crucial factor in the overall score. Contrary to our expectations, the Tzanakis score was not superior for predicting acute appendicitis over the other scores in any of the three age groups in our study. Radiologists carry out US examinations during various working hours; the predictive power of the Tzanakis score will increase if patients are evaluated during daytime working hours by the same experienced radiologist.

The predictive power of the CSSs developed for acute appendicitis varies [1, 27]. The Alvarado scoring system is reportedly more accurate in Western populations, while the RIPASA is more accurate in Middle Eastern and some Asian populations; the two scores are comparable in Eastern populations [16, 28]. The RIPASA score was developed for the patients of RIPAS Hospital, Brunei in 2010. Foreign nationality was added as a variable to this scoring system, given the later hospital admissions of foreign patients (because they generally do not have social security numbers) [28]. Pain tolerance differs between patients of different ethnic origins [29]. The proportion of the immigrant population in our population was 4.37%; furthermore, 45.5% of whom was <20 years of age. No significant difference was found between our patient groups in terms of nationality [30]. This may be one of the reasons why the RIPASA was not superior to the other CSSs in any age group in our study. In addition, the variations of demographic characteristics and socioeconomic levels of immigrants in different societies could explain the inability of RIPASA to outperform other scoring systems in our study.

Gender and negative urinalysis results are only considered in the RIPASA and Ohmann CSSs. Existing pain in the young age group is more likely due to appendicitis. However, in our study, the Ohmann CSS was not superior to any of the other CSSs in any age group. In their 1999 study, Ohmann et al. did not recommend using their CSS as a standard tool for the differential diagnosis of acute appendicitis in any age group [31].

The Fenyo–Lindberg, Lintula, and RIPASA CSSs consider the gender of the patient when predicting acute appendicitis. The Fenyo–Lindberg CSS is more accurate than the others for predicting acute appendicitis in female patients [32]. In our study, the Fenyo–Lindberg CSS was more valuable in the differential diagnosis of acute appendicitis in the 46–65 years group. However, its specificity was low (0.46). It can be concluded that the Fenyo–Linberg scoring system was superior to the others in this age group due to the high female : male ratio in the 46–65 years group (38%).

Various studies have examined the cut-off values to exclude a diagnosis of appendicitis according to the Eskelinen score [33]. The cut-off value was significantly higher in our 18–45 and >65 years age groups than in the 45–65 years group. This may be because right lower quadrant pain is a weighted parameter in the Eskelinen score, and pain tolerance changes with age (Table 4) [20]. In our study, when the cut-off value to exclude appendicitis was 67.7, the Eskelinen CSS was superior to the others in the oldest age group. Lintula et al. developed a scoring system based on examinations of children aged 4–15 years who presented to Kuopio University Hospital with suspected acute appendicitis [18]. Although their scoring system was more accurate in the 18–45 years age group in this study, it was not superior to the other scoring systems.

Muscular defense is the most critical factor affecting the total AIR score. However, the classification of muscular defense as mild, moderate, or high is based on subjective opinions and may differ among clinicians [16]. Considering that muscular defense is weaker during the early stage of the disease, and increases in the later period, the AIR score should be more accurate in elderly patients admitted to hospital in an advanced stage of the disease. However, in our study, the AIRS was not superior in any age group. This may be due to subjective judgments of the severity of examination findings by the surgeons who performed the physical examinations.

Karaman et al. conducted a study in our city in 2018 and stated that the Karaman scoring system, which consists of six parameters, is more accurate for predicting appendicitis than the Alvarado score. However, in our study, the Karaman CSS was not superior to the other scoring systems in any age group [15]. The relatively small sample size of our study group may be the reason why Karaman's score was not found to be superior to other scores among age groups. The results obtained by Karaman et al. and the results obtained in our study are different despite both studies being carried out in the same country. This difference shows that the scoring systems whose validity and reliability have been revealed by various well designed studies should be preferred when choosing the appendicitis scoring system for the diagnosis of acute appendicitis. Almost all novel CSSs are compared to the Alvarado score, as it was the first CSS developed for acute appendicitis and has frequently been shown to be accurate [1, 15, 28, 31, 34, 35]. In our study, the most effective CSS in the 18–45 years age group was the Alvarado score, which was also the second most accurate scoring system (after the Fenyo–Lindberg CSS) among patients of all ages.

### 4.1. Limitations

The main limitation of this study was the small number of patients, particularly in the >65 years age group. Also, this was a single-center study and had a very high number of positive results that inflated the predictive values.

## 5. Conclusion

Appendicitis scoring systems help clinicians make a differential diagnosis in cases where imaging methods cannot be used or are insufficient. In this study, the most accurate scoring system for the differential diagnosis of appendicitis was the Alvarado for the 18–45 years age group and Fenyo–Lindberg CSS for the 46–65 years group. The Eskelinen scoring system was superior to the others in patients aged >65 years; however, it may not be appropriate to use this scoring system in this age group, based on the confidence intervals calculated herein.

## Figures and Tables

**Table 1:** Variables used in scoring systems.

	Alv	Rip	Tza	AIRS	Esk	Ohm	Lint	Fen	Krm
CRP				+					
WBC	+	+	+	+	+	+		+	+
PMNL				+					+
Appendicitis in USG			+						
Nationality		+							
Gender		+					+	+	
Age		+				+			
Pain RLQ		+		+	+	+	+		
Pain level							+		
Pain else RLQ								+	
Pain progression								+	
Migration of pain to the RLQ	+	+				+	+	+	+
Nausea, vomiting	+	+		+			+	+	
Loss of appetite, anorexia	+	+							+
Duration of complaints		+			+			+	
İncreasing pain with cough								+	+
Rigidity, defense		+		+	+	+	+	+	
RLQ tenderness	+	+	+		+	+			
Rebound tenderness	+	+	+	+		+	+	+	+
Rovsing sign		+							
Fever	+	+		+			+		
Leucocyte left shift (>%75 neu)	+								
Absent tinkling or high-pitched bowel sounds							+		
Negative urine analysis. Absence of blood, WBC, bacteria)		+				+			

Alv: Alvarado score, Rip: Ripasa score, Tza: Tzanakis score, AIRS: appendicitis inflammatory response score, Esk: Eskelinen score, Ohm: Ohmann score, Lint: Lintula score, Fen: Fenyo-Lindberg score, Krm: Karaman score. CRP: C-reactive protein, WBC: white blood cell, PMNL: polymorphonuclear leukocyte, USG: ultrasound imaging, RLQ: right lower quadrant.

**Table 2:** Distributions of variables regarding appendicitis in each age group.

		All patients		18–45 years old		46–65 years old		>65 years old	
		App.	Without app.	App.	Without app.	App.	Without app.	App.	Without app.
Gender	Male	118 (91.5)	11 (8.5%)	85 (90.4%)	9 (9.6%)	20 (19.8%)	1 ((4.8%)	13 (92.9%)	1 (7.1%)
	Female	62 (83.8%)	12 (16.2%)	45 (81.8%)	10 (18.2%)	12 (92.3%)	1 (7.7%)	5 (83.3%)	1 (16.7%)
	*p* value	0.09		0.12		0.72		0.5	

Nationality	Native	176 (89.3%)	21 (10.7%)	127 (88.2%)	17 (11.8%)	31 (93.9%)	2 (6.1%)	18 (90%)	2 (10%)
	Foreign	4 (66.7%)	2 (33.3%)	3 (60%)	2 (40%)	1 (100%)	0 (0%)	0	0
	*p* value	0.08		0.06		0.80		0.62	

Fewer	No	169 (88%)	23 (12%)	122 (86.5%9	19 (13.5%)	31 (93.9%)	2 (6.1%)	16 (88.9%)	2 (1.1%)
	Yes	11 (100%)	0 (0%)	8 (0%)	0 (0%)	1 (100%)	0 (0%)	2 (100%)	0 (0%)
	*p* value	0.22		0.26		0.80		0.62	

Right lower quadrant pain	No	5 (83.3%)	1 (16.7%)	2 (66.7%)	1 (33.3%)	2 (100%)	0 (0%)	1 (100%)	0 (0%)
	Yes	175 (88.8%)	22 (11.2%)	128 (87.7%)	18 (12.3%)	30 (93.8%)	2 (6.3%)	17 (89.5%)	2 (10.5%)
	*p* value			0.28		0.72		0.73	

Severity of the pain	Mild	32 (86.5%)	5 (13.5%)	26 (86.7%)	4 (13.3%)	5 (83.3%)	1 (16.7%)	1 (100%)	0 (0%)
	Moderate	83 (87.4%)	12 (12.6%)	57 (85.1%)	10 (14.9%)	18 (94.7%)	1 (5.3%)	8 (88.9%)	1 (11.1%)
	High	65 (91.5%)	6 (8.5%)	47 (90.4%)	5 (9.6%)	9 (100%)	0 (0%)	9 (90%)	1 (10%)
	*p* value	0.63		0.68		0.39		0.94	

Pain outside the right lower quadrant	No	133 (89.3%)	16 (10.7%)	99 (87.6%)	14 (12.4%)	25 (96.2%)	1 (3.8%)	9(90%)	1 (10%)
	Yes	47 (87%)	7 (13%)	31 (86.1%)	5 (13.9%)	7 (87.5%)	1 (12.5%)	9 (90)	1 (10%)
	*p* value	0.66		0.81		0.36		1	

Increasing pain	No	92 (87.6%)	13 (12.4%)	69 (86.3%)	11 (13.8%)	16 (88.9%)	2 (11.1%)	7 (100%)	0 (0%)
	Yes	88 (89.8%)	10 (10.2%)	61 (88.4%)	8 (11.6%)	16 (100%)	0(0%)	11 (84.6%)	2 (15.4%)
	*p* value	0.62		0.69		0.17		0.27	

Pain transition from umbilicus to lower right quadrant	No	78 (83.9%)	15 (16.1%)	53 (81.5%)	12 (18.5%)	12 (93.8%)	1 (7.7%)	13 (86.7%)	2 (13.3%)
	Yes	102 (92.7%)	8 (7.3%)	77 (91.7%)	7 (8.3%)	20 (95.2%)	1 (4.8%)	5 (100%)	0 (0%)
	*p* value	0.047		0.06		0.72		0.39	

Vomiting	No	107 (86.3%)	17 (13.7%)	72 (82.8%)	15 (17.2%)	24 (96%)	1 (4%)	11 (91.7%)	1 (8.3%)
	Yes	73 (92.4)	6 (7.6%)	58 (93.5%)	4 (6.5%)	8 (88.9%)	1 (11.1%)	7 (87.5%)	1 (12.5%)
	*p* value	0.18		0.05		0.43		0.76	

Loss of appetite	No	49 (83.1%)	10 (16.9%)	33 (80.5%)	8 (19.5%)	10 (90.9%)	1 (9.1%)	6 (85.7%)	1 (14.3%)
	Yes	131 (91%)	13 (9%)	97 (89.8%)	11 (10.2%)	22 (95.7%)	1 (4.3%)	12 (92.3%)	1 (7.7%)
	*p* value	0.10		0.12		0.58		0.23	

Duration of symptoms (hours)	<24	94 (87%)	14 (13%)	73 (84.9%)	13 (15.1%)	13 (92.9%)	1 (7.1%)	8 (100%)	0 (100)
	24–48	45 (90%)	5 (10%)	34 (89.5%)	4 (10.5%)	6 (85.7%)	1 (14.3%)	5 (100%)	0 (100)
	>48	41 (91.1%)	4 (8.9%)	23 (92%)	2 (8%)	13 (100%)	0 (0%)	5 (71.4%)	2 (28.6%)
	*p* value	0.73		0.57		0.41		0.12	

Right lower quadrant pain with coughing	No	57 (87.7%)	8 (12.3%)	39 (84.8%)	7 (15.2%)	12 (92.3%)	1 (7.7%)	6 (100%)	0 (0%)
	Yes	123 (89.1%)	15 (10.9%)	91 (88.3%)	12 (11.7%)	20 (95.2%)	1 (4.8%)	17 (85.7%)	2 (14.3%)
	*p* value	0.76		0.54		0.72		0.33	

Bowel sounds with auscultation	None	19 (95%)	1 (5%)	15 (100%)	0 (0%)	3 (100%)	0 (0%)	1 (50%)	1 (50%)
	Normal	156 (89.1%)	19 (10.9%)	111 (87.4%)	16 (12.6%)	28 (93.3%)	2 (6.7%)	17 (94.4%)	1 (5.6%)
	Hyperactive	5 (62.5%)	3 (37.5%)	4 (57.1%)	3 (42.9%)	1 (100%)	0 (0%)		
	*p* value	0.04		0.2		0.86		0.47	

Tenderness in right lower quadrant	No	6 (85.7%)	1 (14.3%)	3 (75%)	1 (25%)	2 (100%)	0 (0%)	1 (100%)	0 (0%)
	Yes	174 (88.8%)	22 (11.2%)	127 (87.6%)	18 (12.4%)	30 (93.8%)	2 (6.3%)	17 (89.5%)	2 (10.5%)
	*p* value	0.80		0.45		0.71		0.73	

Rebound	No	41 (87.2%)	6 (12.8%)	30 (83.3%)	6 (16.7%)	7 (100%)	0 (0%)	4 (100%)	0 (0%)
	Yes	139 (89.1%)	17 (10.9%)	100 (88.5%)	13 (11.5%)	25 (92.6%)	2 (7.4%)	14 (87.5%)	2 (12.5%)
	*p* value	0.72		0.42		0.45		0.45	

Rigidity	None	30 (81.1%)	7 (18.9%)	23 (76.7%)	7 (23.3%)	5 (100%)	0 (0%)	2 (100%)	0 (0%)
	Mild	29 (93.5%)	2 (6.5%)	23 (95.8%)	1 (4.2%)	5 (83.3%)	1 (16.7%)	1 (100%)	0 (0%)
	Moderate	74 (87.1%)	11 (12.9%)	52 (85.2%)	9 (14.8%)	15 (93.8%)	1 (6.3%)	7 (87.5%)	1 (12.5%)
	High	47 (94.0)	3 (6%)	32 (94.1%)	2 (5.9%)	7 (100%)	0 (0%)	8 (88.9%)	1 (11.1%)
	*p* value	0.21		0.09		0.56		0.94	

Rovsing sign	No	111 (87.4%)	16 (12.6%)	79 (84.9%)	14 (15.1%)	22 (95.7%)	1 (4.3%)	10 (90%)	1 (10%)
	Yes	69 (90.8%)	7 (9.2%)	51 (91.1%)	5 (8.9%)	10 (90.9%)	1 (9.1%)	8 (88.9%)	1 (11.1%)
	*p* value	0.46		0.28		0.58		0.88	

App. in USG	No	11 (61.1%)	7 (38.9%)	7 (53.8%)	6 (46.%)	3 (100%)	0 (0%)	1 (50%)	1 (50%)
	Yes	169 (91.4%)	16 (8.6%)	123 (90.4%)	13 (9.6%)	29 (93.5%)	2 (6.5%)	17 (94.4%)	1 (5.6%)
	*p* value	0.00		0.00		0.65		0.04	

Negative urine analysis	No	11 (84.6%)	2 (15.4%)	8 (80%)	2 (20%)	2 (100%)	0 (0%)	1 (100%)	0 (0%)
	Yes	169 (88.9%)	21 (11.1%)	122 (87.8%)	17 (12.2%)	30 (93.8%)	2 (6.3%)	17 (89.5%)	2 (10.5%)

CRP		23.1 ± 76.1	44.2 ± 73.9	18.8 ± 67.8	27.7 ± 57.6	32.8 ± 101.6	111.7 ± 31.4	74.8 ± 68.4	219.2 ± 37.8
	*p* value	0.48		0.83		0.30		0.04	

Leukocyte count		14485 ± 17677	13100 ± 3408	14950 ± 19751	12800 ± 3248	13800 ± 11692	10345 ± 4320	10700 ± 5134	16250 ± 2757
	*p* value	0.05		0.01		0.21		0.16	

App: appendicitis, CT: computerised tomography, CRP: C-reactive protein.

**Table 3:** Distributions of variables for age groups.

Variables		Age groups			*p* value
		18–45 (*n* = 149)	46–65 (*n* = 34)	65+ (*n* = 20)	18–45 (*n* = 149)
Gender	Male	94 (63.1%)	21 (61.8%)	14 (70%)	0.811
	Female	55 (36.9%)	13 (38.2%)	6 (30%)	
Nationality	Native	144 (96.6%)	33 (97.1%)	20 (100%)	0.851
	Foreign	5 (3.4%)	1 (2.9%)	0 (0%)	
C-reactive protein		20.09 (6.04–71.95)	47 (12.13–47)	86.8 (42.6–146.13)	**0.002**
Leukocyte count		14600 (11100–17200)	13600 (11100–13600)	11150 (6380–15200)	**0.049**
Polymorphonuclear leukocyte ratio		78.4 (68–85.1)	80.75 (71.2–80.75)	76.25 (69.75–84.35)	0.692
Left shift in neutrophils	No	92 (61.7%)	16 (47.1%)	12 (60%)	0.303
	Yes	57 (38.3%)	18 (52.9%)	8 (40%)	
Negative urine analysis	No	10 (6.7%)	2 (5.9%)	1 (5%)	1
	Yes	139 (93.3%)	32 (94.1%)	19 (95%)	
Appendicitis in ultrasound imaging	Yes	136 (91.3%)	31 (91.2%)	18 (90%)	1
	No	13 (8.7%)	3 (8.8%)	2 (10%)	
Right lower quadrant pain	Yes	146 (98%)	32 (94.1%)	19 (95%)	0.386
	No	3 (2%)	2 (5.9%)	1 (5%)	
Severity of the pain	Mild	30 (20.1%)	6 (17.6%)	1 (5%)	0.297
	Moderate	67 (45%)	19 (55.9%)	9 (45%)	
	High	52 (34.9%)	9 (26.5%)	10 (50%)	
Pain outside the right lower quadrant	No	113 (75.8%)	26 (76.5%)	10 (50%)	0.05
	Yes	36 (24.2%)	8 (23.5%)	10 (50%)	
Increasing pain	No	80 (53.7%)	18 (52.9%)	7 (35%)	0.322
	Yes	69 (46.3%)	16 (47.1%)	13 (65%)	
Pain transition from umbilicus to lower right quadrant	No	65 (43.6%)	13 (38.2%)	15 (75%)	**0.02**
	Yes	84 (56.4%)	21 (61.8%)	5 (25%)	
Vomiting	No	87 (58.4%)	25 (73.5%)	12 (60%)	0.271
	Yes	62 (41.6%)	9 (26.5%)	8 (40%)	
Loss of appetite	No	41 (27.5%)	11 (32.4%)	7 (35%)	0.737
	Yes	108 (72.5%)	23 (67.6%)	13 (65%)	
Duration of symptoms	<24 hours	86 (57.7%)	14 (41.2%)	8 (40%)	**0.042**
	24–48 hours	38 (25.5%)	7 (20.6%)	5 (25%)	
	>48 hours	25 (16.8%)	13 (38.2%)	7 (35%)	
Right lower quadrant pain with coughing	No	46 (30.9%)	13 (38.2%)	6 (30%)	0.658
	Yes	103 (69.1%)	21 (61.8%)	14 (70%)	
Bowel sounds with auscultation	None	15 (10.1%)	3 (8.8%)	2 (10%)	0.9
	Normal	127 (85.2%)	30 (88.2%)	18 (90%)	
	Hyperactive	7 (4.7%)	1 (2.9%)	0 (0%)	
Tenderness in right lower quadrant	No	4 (2.7%)	2 (5.9%)	1 (5%)	0.663
	Yes	145 (97.3%)	32 (94.1%)	19 (95%)	
Rebound	No	36 (24.2%)	7 (20.6%)	4 (20%)	0.889
	Yes	113 (75.8%)	27 (79.4%)	16 (80%)	
Rigidity	None	30 (20.1%)	5 (14.7%)	2 (10%)	0.333
	Mild	24 (16.1%)	6 (17.6%)	1 (5%)	
	Moderate	61 (40.9%)	16 (47.1%)	8 (40%)	
	High	34 (22.8%)	7 (20.6%)	9 (45%)	
Rovsing sign	No	93 (62.4%)	23 (67.6%)	11 (55%)	0.657
	Yes	56 (37.6%)	11 (32.4%)	9 (45%)	
Fewer	No	141 (94.6%)	33 (97.1%)	18 (90%)	0.624
	Yes	8 (5.4%)	1 (2.9%)	2 (10%)	
Pathology	Acute appandicitis	130 (87.2%)	32 (94.1%)	18 (90%)	0.535
	Normal apendix vermiformis	19 (12.8%)	2 (5.9%)	2 (10%)	

**Table 4:** ROC curve analysis.

	AUC	*p* value	PPV (%)	NPV (%)	Sensitivity (%)	Specificity (%)	Cut-off
*18–45-years-old group*							
Karaman score	0.6285	0.08	092	19	61	63	9
Alvarado score	0.6646	0.01	91	29	83	47	6
Ripasa score	0.6536	0.02	92	19	57	68	11
Tzanakis score	0.6377	0.04	91	19	59	63	15
AIRS	0.5971	0.17	9	60	98	15	4
Eskelinen score	0.5534	0.47	89	22	80	37	61.22
Ohmann score	0.6222	0.06	93	17	43	79	16
Lintula score	0.6393	0.04	90	43	94	31	9
Fenyo-Lindberg score	0.6530	0.03	92	21	66	63	−9

*46–65-years-old group*							
Karaman score	0.6250	0.52	100	8	31	100	12
Alvarado score	0.4688	0.93	96	12	78	50	6
Ripasa score	0.2969	0.01	100	8	25	100	11.5
Tzanakis score	0.3125	<0.01	94	0	100	0	6
AIRS	0.3594	0.50	100	6	9	100	10
Eskelinen score	0.2344	<0.01	94	0	100	0	39.68
Ohmann score	0.1563	<0.01	94	0	100	0	2
Lintula score	0.4844	0.93	100	7	19	100	23
Fenyo lindberg score	0.6875	0.40	100	10	47	100	−6

*65+ years-old-group*							
Karaman score	0.4167	0.57	100	12	17	100	12
Alvarado score	0.4861	0.96	93	20	78	50	6
Ripasa score	0.5000	1.00	94	33	89	50	9.5
Tzanakis score	0.5278	0.90	92	14	67	50	12
AIRS	0.2778	0.43	90	0	100	0	5
Eskelinen score	0.6111	0.28	100	18	50	100	67.6
Ohmann score	0.5000	1.00	100	14	33	100	15
Lintula score	0.3611	0.68	92	14	67	50	17
Fenyo lindberg score	0.4861	0.94	100	13	28	100	−3

PPV: positive predictive value. NPV: negative predictive value. AUC: area under curve.

## Data Availability

Access to data is restricted. The data were obtained with the permission of the hospital management and the ethics committee, with the guarantee that they would not be shared with third parties.
